# Autologous Platelet-Rich Plasma Efficacy in the Field of Regenerative Medicine: Product and Quality Control

**DOI:** 10.1155/2021/4672959

**Published:** 2021-07-29

**Authors:** Marius Nicolae Popescu, Mădălina Gabriela Iliescu, Cristina Beiu, Liliana Gabriela Popa, Mara Mădălina Mihai, Mihai Berteanu, Anca Mirela Ionescu

**Affiliations:** ^1^Department of Physical and Rehabilitation Medicine-“Elias” Emergency University Hospital, “Carol Davila” University of Medicine and Pharmacy, 8 Eroii Sanitari Blvd, 050474 Bucharest, Romania; ^2^Faculty of Medicine, ‘Ovidius' University of Constanta, 1 University Alley, Campus-Corp B, 900470 Constanta, Romania; ^3^Department of Oncologic Dermatology-“Elias” Emergency University Hospital, “Carol Davila” University of Medicine and Pharmacy, 8 Eroii Sanitari Blvd, 050474 Bucharest, Romania; ^4^“Carol Davila” University of Medicine and Pharmacy, 8 Eroii Sanitari Blvd, 050474 Bucharest, Romania

## Abstract

Platelet-rich plasma (PRP) has emerged as a significant regenerative therapy used alone or combined mainly with stem cells, autologous fat grafts, hyaluronic acid, and biomaterials in a variety of medical fields, especially in hair regrowth, wound healing, and sports and rehabilitation medicine. However, the results obtained with this biologic therapy are heterogeneous and conflicting. The observed disparities in the effectiveness of PRP therapies may be due to a lack of standardization in blood processing and preparation. This article is aimed at reviewing the main biological parameters that need to be documented for a thorough reporting of quantitative and qualitative characteristics of the PRP injected, to allow a comparison between the quality of samples and the clinically obtained results and advance the efforts towards treatment standardization.

## 1. Introduction

Platelets (PLTs) are multitalented cells that represent a great reservoir of growth factors (GFs) such as vascular endothelial growth factor (VEGF), epidermal growth factor (EGF), fibroblast growth factor (FGF), transforming growth factor- (TGF-) beta, platelet-derived growth factor (PDGF), and insulin-like growth factor (IGF) [1]. All these growth factors are valuable tools in regenerative medicine, due to their different functions and involvement in mechanisms that aim to restore and regenerate human tissue, such as angiogenesis, fibroblasts proliferation, or extracellular matrix development.

PLTs are activated with tissue injury, through exposure to substances such as thrombin and tissue collagen, and activation leads to the release of inflammatory and growth factors, with the potential of initiating and enhancing natural tissue recovery [2]. Platelet-rich plasma (PRP) is an autologous blood-derived biologic therapy, which is reported to deliver supraphysiologic concentrations of growth factors and other signaling molecules locally at the site of tissue injury, thus intensifying the body's healing efforts [3].

Due to its biological properties, this therapy gained huge popularity among a variety of today's medical fields, with the highest level of evidence in hair regrowth [4], wound healing [5], and sports and rehabilitation medicine [6, 7]. But despite its growing popularity, there is a huge controversy whether the theoretical capacity of the PRP therapy to promote and enhance host cellular regeneration does eventually translate into clinical benefit.

There is a growing need to better understand how PRP works and its benefits so that treatments can be optimized and applied appropriately. This article is aimed at reviewing the main issues creating the gaps between the theoretical effects of PRP therapy and the conflicting clinical results obtained in clinical practice.

## 2. PRP Use in Hair Regrowth, Wound Healing, and Sports and Rehabilitation Medicine

### 2.1. Hair Regrowth

In the past years, accumulating data have shown that PRP may represent a valid regenerative strategy for hair regrowth.

In 2014, Cervelli et al. were the first to perform a histomorphometric analysis on the results obtained by three cycles of injections with autologous activated platelet-rich plasma (AA-PRP) in patients affected by androgenetic alopecia, a progressive and chronic hair loss disorder. It was shown that PRP injections increase the thickness of epidermis and the number of follicles of hair skin, improve the blood supply around the hair follicles, and increase the proliferation of epidermis basal cells and hair follicular bulge cells, thus promoting hair regeneration in androgenetic alopecia [8].

In a randomized, controlled trial published in 2017, Gentile et al. compared the effects of nonactivated PRP versus calcium-activated PRP in hair loss treatment, and both options have proved similar hair density improvements, despite the higher concentration of growth factors (PDGF-BB, TGF-*β*1, and VEGF) depicted in the activated PRP [9]. In the same paper, the authors introduced the possibility to inject the PRP by using a medical injector gun, to precisely control both the delivered dose and the depth of the injection [9, 10].

In 2017, Gentile et al. also published the first paper about the clinical use of autologous micrografts enriched with human hair follicle stem cells (HFSCs), without enzymatic digestion, for the treatment of androgenetic alopecia and hair loss [11]. The reservoir for adult stem cells in this study was the bulge, which is highly rich in epithelial and melanocytic stem cells. The simple centrifugation of the bulb obtained by two millimeters of punch biopsies from the scalp of the patients lead to the development of a liquid suspension enriched with autologous unexpanded human follicle stem cells. The suspension was later injected into the scalp areas affected by hair loss and showed an up to 29% improvement in the hair density for the treated area and less than a 1% improvement in hair density for the placebo area [11].

Extremely interesting, the results of a recent study by Gentile et al. [12] showed that autologous human follicle mesenchymal stem cells (HF-MSCs) and nonactivated PRP (A-PRP) therapy have similar effects on the treatment of androgenetic alopecia: the study detected a hair density improvement of 29.0 ± 5.0% hairs/cm^2^ after the second infiltration for the HFSC treatment group and an improvement of 28 ± 2% hairs/cm^2^ after the third infiltration in patients treated with A-PRP.

Molecular pathways mediating these clinical effects are not yet fully elucidated. It is known that enhancement of Wnt signaling in dermal papilla cells plays a central role in increasing hair regrowth [13]. Mesenchymal stem cells and PRP therapies seem to promote hair growth mainly by suppressing the release and activation of apoptotic proteins such as Bcl-2 and Akt [14]. In addition, these biological therapies increase the expression of fibroblast growth factor 7 (FGF-7) [15], activate extracellular signal-regulated kinase (ERK) [16], and increase Wnt/*β*-catenin signaling [17], leading to accelerated cell growth, prolonged anagen phase of hair follicles, and new hair follicles development.

Nevertheless, in a recently published systematic review, both activated and nonactivated PRP were reported to be a safe and effective alternative treatment for hair loss, when compared with conventional therapies such as topical minoxidil or oral 5-alpha reductase inhibitors (dutasteride, finasteride) [18].

### 2.2. Wound Healing

In the last decade, an exponentially increase has been noticed in the number of clinical trials evaluating PRP therapeutic effects on wound healing and regeneration of soft tissue defects, when used alone or in combination with hyaluronic acid (HA), biomaterials, and fat grafts [19].

The efficacy of PRP used alone for wound healing has been largely reported [20, 21], and in a recently paper by Gentile et al. [22], it was highlighted that each one of the GFs contained in PRP preparations is involved in a specific biomolecular pathway during the healing process of chronic wounds. Furthermore, in an *in vitro* and *in vivo* evaluation, De Angelis et al. [23] reported that combining PRP and HA in a biofunctionalized scaffold caused significant reepithelialization (96.8% ± 1.5% reepithelialization) of chronic diabetic and vascular ulcers, compared to traditional HA dressings alone (78.4% ± 4.4%) within 30 days. Another combination widely investigated in clinical practice is the use of PRP mixed with fat graft and adipose tissue-derived stem cells (AD-MSCs), which has shown promising results in promoting and accelerating the healing process of chronic dermal wounds and posttraumatic extremity ulcers [24].

### 2.3. Sports and Rehabilitation Medicine

In these fields, a number of injectable agents, including glucocorticoids [25], hyaluronic acid derivatives [26], and botulinum toxin [27], have been used for the treatment of various musculoskeletal conditions. In the latest years, platelet-rich plasma therapy has been widely popularized for the local treatment of soft-tissue and musculoskeletal injuries such as osteoarthritis, ligament injuries, muscle tears, and tendinopathies [28].

However, despite the amount of available data to support the use of PRP in the field of regenerative medicine, this treatment method lacks high-quality evidence [29]. Only a small number of controlled trials support its use, whereas the majority of the clinical trials of PRP lack high-quality evidence of the efficacy of PRP treatments and have small sample sizes or high risk of bias [29].

Also, in the available clinical trials, in most of the cases, the PRP obtained product is not properly characterized, and interstudy comparability is limited. PRP is a general denomination describing a therapy that is highly heterogeneous in preparation techniques. This inconsistency leads to a range of variations in the concentration of active substances in the product that has to be injected and therefore may change the biological features and benefits of PRP [30].

## 3. The Variety of Materials Used for Blood Harvesting Techniques

For the available PRP commercial systems, blood can be collected from the patients with the use of a variety of techniques as follows:

- Vacuum blood-collection tubes containing anticoagulants that may be plain tubes or may contain a separating gel that separates the red blood cells from platelets and plasma at the end of the centrifugation process
- Anticoagulant prefilled syringes that can further undergo immediate centrifugation or may be transferred either in a secondary disposable or in an automated device for centrifugation process thus obtaining the final product to inject
- Blood-collection bags prefilled with anticoagulant

In addition to the different techniques used for blood harvesting, these devices are completely different based on the anticoagulant that is used, the volume, the numbers, the times and the speed of centrifugation, removal or not of the platelet-poor plasma (PPP) part, or the need to resuspend the PLTs into the manual devices [22]. Therefore, it is predictable that each device can produce different biological PRP product.

## 4. Systematic Biological Characterization of the Injected PRP Is Lacking

Maxillofacial surgeon Robert Marx was the first to use PLTs in this field, using a basic clear definition: “PRP is defined as a suspension of platelets in plasma characterized by a platelet concentration which is higher than the concentration of the original blood collected” [31]. This pioneer publication offered a lot of details about the preparation of PRP sample, about platelets counting for each patient, about the isolated growth factors, and provided a very informative conclusion that for autologous plasma to have high healing properties for bone and soft tissue; the platelet levels should reach the concentration of 1,000 × 10^9^/L in 5 mL of plasma.

Beginning with this paper, a growing interest in PRP for therapeutics has been illustrated by the rapid growth in publications on this topic, with over 500 clinical trials relating to “platelet rich plasma” listed on clinicaltrials.gov (March 2021). The number of randomized clinical trials is increasing each year, but there is one big weakness: in most cases, no characterization of the PRP product is available.

We have herein investigated and synthesized the main variables that need to be documented for a thorough analysis of PRP samples (Figure 1).

### 4.1. The Volume of PRP

This needs to be specified since it is directly affecting the concentration.

### 4.2. Platelets Increase Factor

The platelet increase factor refers to the platelet concentration increase in PRP product compared with native peripheral blood, and it is thought to primarily influence the PRP efficacy. Manufactures are largely emphasizing that higher platelet increase factor directly correlates with higher PRP efficacy, but this is only partially true. A platelet concentration in PRP lower than in native peripheral blood may be indeed suboptimal and inefficient but, however, too high platelet concentrations (sixfold higher than baseline) may induce an inhibitory effect on osteoblast activity and healing processes [32].

### 4.3. Leukocytes Increase Factor

In 2009, Dohan Ehrenfest et al. [33] introduced the concept of leukocyte-rich PRP (LR-PRP), characterized by a total white blood cell (WBC) count higher than the WBC level in the native blood, versus leukocyte-poor PRP (LP-PRP), which is characterized by a total WBC count lower than the WBC level in native blood.

The concentration of leukocytes (which contain enzymes such as collagenase) could have a different impact on cartilage and tendon cells. The results of a meta-analysis of randomized trials suggest that LR-PRP may be more effective than LP-PRP for the treatment of tendinopathies [4].

A recent systematic review and meta-analysis of available studies regarding treatment of knee osteoarthritis also indicated that LR-PRP has more proinflammatory properties than LP-PRP [34].

### 4.4. Dose of Injected Platelets (Concentration (PLTs) × Volume)

In 2016, Magalon et al. analyzed 20 PRP preparations and concluded that the dose of injected platelets can vary from 0.21 to 5.43 billion, depending on the device used, meaning that the increased fold between two devices can vary by more than 25-fold, and therefore, it is perfectly understandable that the therapeutic effects may be different [35]. A positive correlation between the platelet dose and the quantity of growth factors delivered at the injections site has been shown in this paper, as well as in previous studies.

### 4.5. The Global and Relative Composition of the PRP

This refers to the characterization of PRP preparations, by their concentration of PLTs, leukocytes, and red blood cells (RBCs).

One of the most important concerns in PRP products is the detection of the level of RBCs contamination, an aspect that is otherwise not included in the current classifications of PRP. It has been shown that a great number of PRP preparation devices provide more RBCs than PLTs in the final PRP product [36]. The degradation processes of RBCs present in the PRP preparation generate pathophysiological processes including hemolysis and eryptosis, with potential consequences such as inflammation, radical oxygen reactions, cellular stress, vasoconstriction, and impaired cell metabolism, thus impeding the beneficial action of PRP [37].

Furthermore, in sports medicine, an *in vitro* stud*y* performed on human synovial cells showed that using PRP rich in erythrocytes and leukocytes promotes synoviocyte cell death and proinflammatory mediator production, which could lead to intra-articular injury [38].

### 4.6. The Capacity of the Device to Recover All the Platelets from the Blood (the Recovery Rate in Platelets)

This parameter refers to the percentage of PLTs captured in the PRP from initial whole blood. It is not directly correlated to clinical efficacy, but it is rather an indicator of the performance of the PRP preparation device and is currently used only in DEPA classification [36].

In various studies, the recovery rates in PLTs for several devices ranged from 13.1% [39] to 79.3% [40]. In a recent 2021 technical and biological analysis of authorized medical devices for platelet-rich plasma preparation, Magalon et al. [41] found that these systems still fail to recover approximately 40% of the platelets from the blood during the preparation step (the mean recovery rate in PLTs is approximately 60%). Furthermore, most of the preparations that did manage to achieve a recovery rate higher than 80% also presented a high rate of RBC contamination, highlighting that the available centrifugation cycles are not yet capable of reaching both PRP purity and high recovery rate of PLTs.

### 4.7. Activation Process

Activation is required for platelets to degranulate and release bioactive molecules [42, 43].

To this regard, before injecting PRP into the target tissue, exogenous platelet activators can be added, such as calcium chloride, thrombin, or collagen. On the other hand, some authors state that PRP products can be used without the addition of an activation agent because platelet activation is spontaneously induced due to exposure to dermal collagen and thrombin once PRP is injected [9, 44].

The issue concerning the need for exogenous activating substance is controversial but is important for clinicians to always specify the activation status since different PRP activation agents can affect the physical form of the final product and might also influence the release curve of growth factors.

## 5. International Biological Classifications Designed to Define PRP Need to Be Implemented in Clinical Practice

In the late years, a lot of international scientific societies with interest in advancing PRP therapies have issued recommendations to optimize and standardize the use of PRP products, and seven different biological classification systems are currently available to simplify the use of PRP: the Paw Classification system [43], the Mishra classification system [42], PLRA classification [45], DEPA classification [36], MARSPILL classification [46], the ISTH classification [47], and AAOS edited consensus recommendations [48].

These classifications assess different biological parameters and have different thresholds concerning the concentration of PLTs in the whole blood, the global and relative composition (PLTs, leukocytes, and RBCs) of the PRP, cells increased or decreased factors compared to blood, the dose of injected PLTs, and the remaining percentage of PLTs in PRP from initial whole blood (recovery rate in platelets). But most importantly, overall, all these classifications clearly state that to correctly classify PRP, a cell count is implied both for the blood and the PRP samples.

One of the latest recommendations is issued by the Platelet Physiology Subcommittee of the Scientific and Standardization Committee (SSC) of the International Society on Thrombosis and Haemostasis (ISTH), which highlights the need to take into account the content and the quality control of the platelet preparation to ensure that clear correlation can be established between the biological quality and the clinical outcomes [47].

The consensus recommendations edited by the American Academy of Orthopaedic Surgeons (AAOS) are further providing minimum standards for product development and clinical research evaluating PRP, with no less than 23 parameters that need to be reported in clinical trials, to allow for reproducibility and comparison across studies. The same prestigious scientific society recommended that physicians and institutions offering PRP biologic therapies should establish postmarket monitoring and quality assessments, by using high-quality biorepository-linked registries [48].

Implementation of all these classifications and recommendations is very important, but, unfortunately, they are still not adopted in clinical practice.

This is mainly because in real life practice such systematic biological characterization is expensive and time consuming. It requires access to an automatic cell counter or a collaborative work with a medical laboratory and access to a performant software that would further allow exploitation of the generated data by qualified staff. Very few physicians manage to achieve this at an individual level, and in the future development of Centers of Excellence in Regenerative Medicine could allow a homogenization of the practices and empower follow-up of international recommendations.

## 6. Conclusions

Autologous platelet-rich plasma therapy describes a treatment without standardization of manufacturing process and guidelines of use, and thus, the evidence for its efficacy is conflicting and limited in quality. The differences detected in the effectiveness of this biologic therapy may be caused by the wide disparities in PRP preparation and a lack of standardization in blood processing methods. Validation of this therapy will demand further standardization of PRP preparation methods for clinical use, with a focus on the quantitative and qualitative characteristics of the injected PRP.

## Figures and Tables

**Figure 1:** Biological parameters that need to be evaluated for a proper analysis of the platelet-rich plasma (PRP) preparations.
